# Micro-RNAs as diagnostic or prognostic markers in human epithelial malignancies

**DOI:** 10.1186/1471-2407-11-500

**Published:** 2011-11-30

**Authors:** Angela Hui, Christine How, Emma Ito, Fei-Fei Liu

**Affiliations:** 1 Ontario Cancer Institute (OCI)/Campbell Family Cancer Research Institute (CFCRI); University Health Network (UHN); Toronto, ON, Canada; 2 Department of Medical Biophysics; University of Toronto; Toronto, ON, Canada; 3 Department of Radiation Oncology; Princess Margaret Hospital; UHN; Toronto, ON, Canada; 4 Department of Radiation Oncology; University of Toronto; Toronto, ON, Canada

## Abstract

Micro-RNAs (miRs) are important regulators of mRNA and protein expression; the ability of miR expression profilings to distinguish different cancer types and classify their sub-types has been well-described. They also represent a novel biological entity with potential value as tumour biomarkers, which can improve diagnosis, prognosis, and monitoring of treatment response for human cancers. This endeavour has been greatly facilitated by the stability of miRs in formalin-fixed paraffin-embedded (FFPE) tissues, and their detection in circulation. This review will summarize some of the key dysregulated miRs described to date in human epithelial malignancies, and their potential value as molecular bio-markers in FFPE tissues and blood samples. There remain many challenges in this domain, however, with the evolution of different platforms, the complexities of normalizing miR profiling data, and the importance of evaluating sufficiently-powered training and validation cohorts. Nonetheless, well-conducted miR profiling studies should contribute important insights into the molecular aberrations driving human cancer development and progression.

## Introduction

Micro-RNAs (miRs) are important regulators of mRNA and protein expression which play important yet complex roles in human cancers [1]. Their biogenesis and biological networks are complex (Figure 1); they are first synthesized as large RNA precursors, processed in the nucleus into approximately 70 nt pre-miRs, folded into imperfect stem-loop structures, transported to the cytoplasm, whereupon they are incorporated into RISC (RNA-induced silencing complex) (reviewed in [2]). Cleavage by Argonaute-2, then Dicer, results in an approximately 22-nt mature miR duplex; the "guide" strand is retained within the RISC; the "passenger" strand is degraded. Through the seed region (nt 2 to 8), the miR can then bind to the 3'UTR of target mRNA sequences, preventing protein translation, leading to mRNA degradation. More recently, miRs have also been described to target 5'UTR, and even coding regions of transcripts [3]. The current miRDatabase (http://www.mirbase.org) has catalogued more than 1,300 human sequences. Given their ability to target mRNA with imperfect complementarity, and predicted to regulate the expression of approximately one-third of all human transcripts [4], miRs are considered to be among the largest class of gene regulators [5,6].

**Figure 1:** **Micro-RNA biogenesis**. MiR's are synthesized initially as large RNA precursors (pri-miRs), processed in the nucleus by RNAse III Drosha, and DGCR8 into approximately 70 nt pre-miR, which are transported to the cytoplasm by exportin-5, with subsequent cleavage by another RNAse III enzyme Dicer, with its co-factor TRBP, releasing the approximately 22-nt mature dsmiR. MiR's can negatively regulate their targets in one of two major ways, depending on the degree of complementarity to its target. First, and probably most commonly, one strand of this duplex is incorporated into the RNA-induced silencing complex (RISC), then binds with imperfect complementarity to the 3'-UTR (untranslated region) of mRNA targets, preventing protein translation. Alternatively, miRs can bind with perfect complementarity to the ORF (open reading frame) of target mRNA's with subsequent degradation. Recent evidence also indicates miRs can also bind to either promoters, or coding regions of mRNAs as additional mechanisms of regulation.

Multiple mechanisms can mediate miR dysregulations in human cancers, including chromosomal gains or losses [7], mutations of miR located loci [8], or epigenetic aberrations [8]. Any misstep in miR biogenesis (Figure 1) can also affect miR expression [9,10], exemplified by the down-regulation of Drosha and Dicer being associated with worse survival in ovarian, lung, and breast cancers [11]. MiRs can be either over- or under-expressed, functioning as tumour suppressors or oncogenes, depending on their downstream target genes [12]. MiR-15a and miR-16-1 are two of the first described down-regulated miRs in chronic lymphocytic leukemia [13], both target Bcl-2 [14]; thus their absence inhibits apoptosis. Alternatively, miR-21, one of the most commonly over-expressed miRs in solid malignancies, targets PTEN [15] and pro-apoptotic genes [16,17]; hence pro-survival signals dominate.

## Micro-RNA as bio-markers in epithelial cancers

Biomarkers are biological indicators of disease states, utilized to define tumor subtypes, or assess efficacy of interventions [18]. Useful biomarkers can provide insights into tumorigenesis, and facilitate the development of improved therapies. Some current bio-markers include prostate-specific antigen (PSA) [19], carcinoembryonic antigen (CEA) [20], CA125 [21], and α-fetoprotein [22,23]. More recently, the role of mRNA or miRs as cancer biomarkers have also been investigated and developed. The prototype mRNA signature is Oncotype DX, the 21-gene set utilized to predict recurrence risks for patients with breast cancer [24].

MiR expression profilings could distinguish different cancer types [12], classify sub-types of prostate or breast cancers [25], identify the tissue origin of tumors [26], and facilitate the diagnosis of colon [27], or lung cancers [28]. MiRs can also predict outcome, such as let-7a [28] and miR-155 [29] for lung cancer, and select patients for targeted therapy (for example, breast cancer [30]). Finally, predictive miR signatures have been reported for several malignancies, such as lung [31-34], hepatocellular [35], esophageal [36], gastric [37], prostate [38] cervical [39], and colon cancers [40].

### Micro-RNAs in FFPE samples

The ability to examine FFPEspecimens, a universally standard histologic processing procedure, allows the expeditious discovery and evaluation of potential biomarkers, given their possible link to clinical databases with mature follow-up. Transcript (mRNA) profiling is technically challenging with FFPE samples due to significant RNA degradation during formalin fixation [41,42], and continued deterioration with storage over time [43]. In contrast, miRs are not significantly affected by fixation, and can be readily extracted from FFPE samples due to their small sizes (approximately 22 nt in length) and remarkable stability [44,45]. Hence, this greatly enhances the ability to evaluate miRs as cancer biomarkers, leading to a multitude of reports describing miR expressions in many epithelial malignancies, summarized as per anatomical site in Table 1.

**Table 1:** Micro-RNAs as Diagnostic or Prognostic markers in FFPE Samples

Cancer	Diagnostic miRs	Prognostic miRs	References
**Head and Neck Squamous cell carcinoma**	miR-16, -20a, -21, -106b, -142-3p, -155, -423, let-7i (up); miR-10a, -125b, -375 (down)	miR-451 (up)	[47]
			
**Breast cancer**	miR-21(up); let-7a, miR-145, -205 (down)		[70]
		miR-21 (up)	[71]
	miR-21, -155, -191, -196a (up); miR-125b, -221 (down)		[44]
			
**Lung cancer**	miR-21, -205		[72]
		miR-16 (up)	[73]
			
**Gastrointestinal Cancers**			
**Gastric cancer**	miR-106a (up)		[74]
	miR-31 (down)		[75]
		miR-10b, -21, -223, -338 (up); miR-30a-5p, -126, let-7a (down)	[37]
**Pancreatic cancer**	miR-452, -105, -127, -518a-2, -187, -30a-3p (up)	miR-196a-2 (up)	[76]
	miR-21, -155 (up)		[77]
	miR-21, -221, -222, let-7a (up)		[78]
		miR-200c (down)	[79]
			
**Gynecological Cancers**			
**Cervical cancer**		miR-9, -200a	[39]
**Ovarian cancer**		miR-223 (up); miR-9 (down)	[80]
		miR-200a, -200b, -429 (down)	[81]
		miR-23a, -27a (up)	[82]
		miR-29b (up)	[83]
			
**Prostate cancer**	miR-125b (up)		[84]
	miR-15a, -16 (down)		[85]
	miR-184 (up); miR-146a (down)	miR-184 (up)	[86]
	miR-203 (down)		[87]
	miR-34c (down)	miR-34c (down)	[88]
		miR-221 (down)	[89]

As already mentioned, miR-21 up-regulation is the most commonly observed aberrant miR in human cancers, with oncogenic consequences [46] (Table 1). It was first reported in glioblastoma [16], but also described for epithelial cancers such as head and neck, breast, colon, lung, prostate, and others [12,44,47]; often associated with worse outcome [40]. Over-expression of miR-21 has been shown to increase cell proliferation, migration, invasion and survival [48]; in contrast, suppression of miR-21 induced apoptosis and decreased cell proliferation and invasion [49].

Mir-155 is another commonly dysregulated miR, wherein the majority of studies report its over-expression associated with tumorigenesis in lymphomas, breast, lung, colon, pancreatic cancers, and others [50]. Aside from these two miRs, there is usually minimal overlap of dysregulated miRs described amongt different studies, even when examining the same cancer type; the same variation as previously observed for mRNA profiling. Perhaps this might relate to multiple redundant "wirings" in human cancers [51], wherein just as four distinct mRNA profiles can all predict for breast cancer relapse [52], a similar phenomenon might also apply to miR profiles, although this remains to be definitively proven.

### Micro-RNAs in blood samples

There is emerging interest in the investigation of miRs as non-invasive biomarkers in circulating blood. This was first described in B-cell lymphoma, reporting elevated levels of miR-155, -210 and -21 in patients' sera, with miR-21 associating with relapse-free survival [53]. In epithelial cancers, Mitchell *et al*. first identified tumor-derived miRs in plasma samples, and suggested that variations in miR abundance reflected tumor burden [54]. MiRs have been detected as free miRs in either plasma or serum, or contained within microvesicles such as exosomes; the latter being minute, natural membrane vesicles secreted by a variety of different cell types [55]. In addition to miRs, exosomes also carry intact and functional mRNA [56], with the probable purpose of transferring information and signals throughout the body [55]. Association of epithelial cancer and exosome miRs was first illustrated in ovarian cancer, wherein tumor-derived miR profiles strongly correlated with levels of peripheral blood-derived exosomal miRs [57]. Similar observations have also been reported for lung cancer [58,59].

As shown in Table 2, the list of potential blood miR biomarkers is even more diverse than those from tissue studies (Table 1). The greatest degree of overlap was reported for miR-21, miR-196a and miR-210 from four different pancreatic cancer studies [60-63]. As observed for the tissue studies, miR-21 and miR-155 are also the two most common aberrant miRs in circulation with putative diagnostic and prognostic value (Table 2). However, down-regulation of miR-155 was reported in one serum study of ovarian cancer [64]. There is some controversy surrounding miR-155; the majority of reports suggest an oncogenic role; however, in a lung cancer study, its up-regulation predicted for worse outcome for adenocarcinomas, but improved outcome for squamous cell carcinoma patients [65]. One possible tumor suppression function for miR-155 was demonstrated in miR-155 deficient mice, which appeared to reduce oncogenic translocations generated by activation-induced cytidine deaminase (AICD) [66]. Micro-RNA expression levels in circulation can also relate to hormone receptor status in that estrogen negative breast cancer sera samples had higher levels of miR-21 and miR-10b [67]; in contrast. miR-155 was detected for progesterone receptor positive patients [68].

**Table 2:** Micro-RNAs as Non-invasive Biomarkers in Blood Samples

Cancer	Samples	Diagnostic miRs	Prognostic miRs	References
**Head and Neck**	Plasma	miR-184 (up)		[90]
**Squamous cell carcinoma**	Plasma	miR-24 (up)		[91]
	Plasma	miR-31 (up)		[92]
	Plasma	miR-181 (up)	miR-181 (up) correlated with poor survival, lymph-node metastasis, and vascular invasion	[93]
				
**Breast cancer**	Serum		miR-155 (up) in PR+ve patients	[68]
	Plasma	miR-425*(up); let-7d*(down)		[94]
	Serum	miR-10b, -34a, -155 (up)	miR-10b, -34a, -155 (up) correlated with metastasis	[95]
	Serum	miR -21, -106a, -155 (up); miR-126, -199a, -335 (down)		[96]
	Whole blood	miR-195 (up)	miR-21, -10b (up) in ER -ve patients; let-7a (down) in lymph node +ve patients	[97]
	Serum		miR-21 (up) correlated with visceral metastasis	[98]
				
**Non-small-cell lung carcinoma**	Pooled serum	miR-25, -223 (up)		[99]
	Exosome from plasma	miR-17-3p, -21, -106a, -146, -155, -191, -192, -203, -205, -210, -212, -214 (up)		[58]
	Pooled serum		miR-486, -30d (up); miR-1, -499 (down) associated with overall survival	[100]
	Serum	miR-10b, -155 (up)	miR-10b (up) associated with lymph node metastasis	[101]
	Vesicles of plasma samples	let-7d, let-7f, miR-223, -383, -192, -30e-5p, -301, -572, -20b, -345 (down)	let-7f, miR-30e-3p (up) associated with poor outcome	[59]
				
**Gastrointestinal Cancers**				
**Colorectal cancer**	Plasma	miR-17-3p, -92 (up)		[102]
	Plasma	miR-29a, -92a (up)		[103]
	Plasma	miR-221 (up)	miR-221 (up) associated with poor overall survival	[104]
**Esophageal**	Serum	miR-10a, -22, -100, -148b, -223, -133a, -127-3p (up)		[105]
**Gastric cancer**	Serum	miR-1, -20a, -27a, -34, -423-5p (up)	miR-1, -20a, -27a, -34, -423-5p (up)	[106]
	Plasma	miR-17-5p, -21, -106a, -106b (up); let-7a (down)		[107]
**Hepatocellu-lar carcinoma**	Serum	miR-500 (up)		[108]
	Serum	miR-1, -25, -92a, -206, -375, -let-7f (up) (HBV-associated); miR-25, -375, and let-7f (up) (HCC detection)		[109]
	Serum	miR-21, -122, -223 (up)		[110]
	Serum	miR-122 (up)		[111]
	Serum	miR-885-5p (up)		[112]
	Serum	miR-16 (down) combined with AFP, AFP DCP increases specificity of HCC detection		[113]
**Pancreatic cancer**	Plasma	miR-21, -210, -155, -196a (up)		[63]
	Plasma	miR-210 (up)		[62]
	Plasma	miR-21 (up)		[60]
	Serum	miR-21, -155, -196a (up)	miR-196a (up)	[61]
				
**Ovarian cancer**	Exosome from serum	miR-21, -141, -200a, -200c, -200b, -203, -205, -214 (up) correlated with stage	miR-21, -141, -200a, -200c, -200b, -203, -205, -214 (up) correlated with stage	[57]
	Serum	miR-21, -92, -93, -126 -29a (up); miR-155, -127, -99b (down)		[64]
	Whole blood	miR-30c1* (up); miR -342-3p, -181a*, -450b-5p (down)		[114]
				
**Prostate cancer**	Serum	miR-141 (up)	miR-100, -125b, -141, -143, -296 (up)	[54]
	Serum	miR-16, -92a, -103, -107, -197, -34b, -328, -485-3p, -486-5p, -92b, -574-3p, -636, -640, -766, -885-5p (up)		[115]
	Serum	miR-20b, -874, -1274a, -1207-5p, -93, -106a (up); miR- 223, -26b, -30c, -24 (down)	miR-24 (down) in metastatic cancers	[116]
	Serum	miR-375, -141 (up)	miR-375, -141 (up)	[117]
	Serum	miR-21 (up)	miR-21 (up) associated with resistant to docetaxel-based chemotherapy	[118]
	Serum	miR-21, -141, -221 (up)	miR-21, -141, -221 (up)	[119]

In summary, there are multitudes of reports describing the potential value of miRs as both diagnostic and prognostic bio-markers for human malignancies. None to date, however, have been translated into clinical practice, likely a reflection of its complex biology, and lack of validation studies using appropriately-powered sample sizes.

### Challenges of Micro-RNA as bio-markers

Despite the promising data supporting the potential value of miRs as biomarkers, many challenges remain. First, robust platforms, as well as appropriate statistical and bio-computational analyses must be utilized in order to identify potential candidate miR signatures for predicting outcome. Furthermore, such candidate signatures must be validated using independent cohorts statistically powered to confirm the existence of a predictive signature. Second, the selection of the appropriate reference controls is extremely important for normalization of biological variation. Recent reports have observed that some of the commonly-utilized reference miRs, such as RNU43, RNU44 or RNU48, in fact fluctuate with the biological entity of interest [69]; hence it is critical to determine the most stable miRs for each condition under examination. Third, it is conceivable that given the "upstream" effects of miRs, and their biological complexities which we are just starting to unravel, their pattern of expression might be too subtle and variable to serve as robust predictive signatures. Nonetheless, pursuit of investigations such as prognostic signatures, or their measurements in sera/plasma are definitely warranted, particularly when using appropriately-sized population cohorts.

## Conclusion

Application of the potential role of miRs as molecular bio-markers in human epithelial malignancies is widely supported by the large number of studies conducted in different cancers. There is great promise that they will aid in the early diagnosis of cancer, and the development of personalized therapies. Further research into miR biogenesis and regulation, along with functional target identifications will definitely lead to an improved understanding of the complex mechanisms underlying human cancer development and progression.

## Abbreviations

AICD: activation-induced cytidine deaminase; CEA: carcinoembryonic antigen; FFPE: formalin fixed and paraffin embedded; miRs: micro-RNAs; PSA: prostate-specific antigen; RISC: RNA-induced silencing complex.

## Competing interests

FF Liu is a Section Editor for *BMC Cancer*.

## Authors' contributions

AH performed the literature review and prepared the manuscript. CH performed the literature review and participated in manuscript preparation. EI prepared the figure. FL designed and edited the manuscript. All authors read and approved the final manuscript.

## Pre-publication history

The pre-publication history for this paper can be accessed here:

http://www.biomedcentral.com/1471-2407/11/500/prepub
